This article has been retracted.

# W-GPCR Routing Method for Vehicular Ad Hoc Networks

**DOI:** 10.3390/s20123406

**Published:** 2020-06-16

**Authors:** Min Li, Zhiru Gu, Yonghong Long, Xiaohua Shu, Qing Rong, Ziji Ma, Xun Shao

**Affiliations:** 1 College of Traffic Engineering, Hunan University of Technology, Zhuzhou 412007, China; minli0103@126.com (M.L.); lyhcai@126.com (Y.L.); sxhdata@126.com (X.S.); Rong08017@163.com (Q.R.); 2 College of Electrical and Information Engineering, Hunan University, Changsha 410082, China; zijima@hnu.edu.cn; 3 Division of Information and Communication Engineering, Kitami Institute of Technology, Hokkaido 090-8507, Japan; x-shao@ieee.org

**Keywords:** VANET, weight choice, GPSR, GPCR

## Abstract

The high-speed dynamics of nodes and rapid change of network topology in vehicular ad hoc networks (VANETs) pose significant challenges for the design of routing protocols. Because of the unpredictability of VANETs, selecting the appropriate next-hop relay node, which is related to the performance of the routing protocol, is a difficult task. As an effective solution for VANETs, geographic routing has received extensive attention in recent years. The Greedy Perimeter Coordinator Routing (GPCR) protocol is a widely adopted position-based routing protocol. In this paper, to improve the performance in sparse networks, the local optimum, and the routing loop in the GPCR protocol, the Weighted-GPCR (W-GPCR) protocol is proposed. Firstly, the relationship between vehicle node routing and other parameters, such as the Euclidean distance between node pairs, driving direction, and density, is analyzed. Secondly, the composite parameter weighted model is established and the calculation method is designed for the existing routing problems; the weighted parameter ratio is selected adaptively in different scenarios, so as to obtain the optimal next-hop relay node. In order to verify the performance of the W-GPCR method, the proposed method is compared with existing methods, such as the traditional Geographic Perimeter Stateless Routing (GPSR) protocol and GPCR. Results show that this method is superior in terms of the package delivery ratio, end-to-end delay, and average hop count.

## 1. Introduction

Since the advent of the car, driving safety has been a major concern in the field of transportation. Reducing traffic accident casualties usually involves two aspects: reducing the incidence of accidents by installing brake assist and electronic stability control systems in vehicles; and by installing protective equipment, such as seat belts and airbags, in vehicles to reduce the rate of casualties in the event of an accident. The rapid development of in-vehicle sensor technology has led to safety features such as blind-spot detection technology, lane departure detection technology, and forward collision warning technology. These innovations can help reduce the incidence of traffic accidents, but the measurement accuracy and reliability of sensors have certain limitations. Under the influence of severe weather conditions and other force majeure factors, performance will be significantly reduced. In order to solve the shortcomings of sensors, many researchers have investigated Internet of Vehicle (IoV) technology. Using vehicle to vehicle (V2V) and vehicle to road (V2R) communications to exchange information [1] can greatly improve the vehicle’s ability to perceive the surrounding environment and predict accidents, and further reduce the accident rate. V2X (Vehicle to X) technology has become a popular research topic in China and abroad in recent years. V2X is a preventive safety technology, which, in addition to addressing driving safety issues, will also play a significant role in improving traffic efficiency, alleviating congestion, and reducing environmental pollution [2,3].

As an emerging field of MANETs (mobile ad-hoc networks), VANETs (vehicle ad-hoc networks) are a form of wireless communication network, with the purpose of improving driver safety and passenger comfort. A VANET is a wireless network in which nodes are both network participants and collaborators through the wireless communication equipment [4] installed on each node. Nodes communicate through other intermediate nodes within their transmission range to form a network. A VANET is a self-organizing network and does not depend on any fixed network infrastructure. Although some fixed nodes act as roadside units, it is convenient to provide geographical location data for the vehicle network or access to the Internet [5,6]. The high-speed dynamics of the nodes are the main characteristics of VANETs, which also leads to rapid changes in the network topology [7]. In order to provide reliable services, a VANET needs to solve many challenges. Establishing reliable routing is one of the main challenges, so more research is needed to promote the development of VANETs.

Traditional IoV routing protocols are divided into two main types: a topology-based routing protocol, and a location-based routing protocol. The topology-based routing protocol uses the link information in the network to send data packets from the source node to the target node. This method is not suitable for high-speed moving vehicle node networks, because the high-speed mobility of nodes causes the network topology to change rapidly. Depending on the link information in the network, the data packet may not be successfully sent to the target node. Because of the movement of nodes, the amount of routing table information in the network that is updated in real-time is very large, and the network overhead is also very large. As a result, this method does not apply to the current Internet of Vehicles [8].

The location-based routing protocol uses the geographic location information of the nodes to establish a data link from the source node to the target node. It fully adapts to the high-speed dynamic characteristics of vehicle nodes. Unlike topology-based routing protocols, location-based routing protocols do not require any routine maintenance. The protocol only determines a data link when it needs to forward data packets, so the network overhead is small. The above features make the location-based routing protocol more suitable for the Internet of Vehicles.

Location-based routing protocols are divided into the following five main categories:

1. Routing protocols based on greedy algorithms, such as Geographic Perimeter Stateless Routing (GPSR) [9] and Greedy Perimeter Coordinator Routing (GPCR) [10] protocols. When the source node knows the location of its target node, this type of routing protocol greedily chooses to forward the data packet to the neighbor node closer to the target node until the data packet is successfully sent to the target node. When a node forwards data, it does not need to know the status information of nodes other than the target node and neighbor nodes. This reduces the cost of routine maintenance. When forwarding data, there is only one next-hop node selected, and there is no need to flood forward data.
2. Routing protocols based on mobile prediction, such as DGRP (Directional Greedy Routing Protocol) [11], PDGR (Predictive Directional Greedy Routing) [12], PGRP (Predictive Geographic Routing Protocol) [13], and MPBRP (Mobility Prediction Based Routing Protocol) [14]. In this type of routing protocol, the location of the node is predicted. In the selection of nodes, the reference indexes of the movement direction and position of the nodes are weighed. This can reduce the number of routing hops and end-to-end delay. However, this kind of routing needs to predict the position of the current node and all of its neighboring nodes, which increases the calculation task of the system and increases the network overhead.
3. Routing protocols based on delay tolerance, such as GeoDTN+Nav (Geographic Delay Tolerant Network Routing With Navigator) [15]. This type of routing protocol mitigates the impact of network partitions and intermittent connections through a delay-tolerant store-and-forward scheme, thereby improving the reachability of routes. However, this kind of routing protocol has a poor real-time performance. When the data packet is cached to a certain node, and there is no suitable opportunity to forward it, the information will be lost due to the excessive accumulation of data packets.
4. Routing protocols based on a combination of topology and location, such as GPCR-D(A Topology and Position Based Routing Protocol in VANET) [16] and HybTGR (Hybrid Routing Protocol Based on Topological and Geographical) [17]. In this type of routing protocol, each network node is assigned a weight based on parameters including the node’s moving speed, the life of the routing link, the number of vehicles near the node, and the distance to the target node. According to the weight, the topology or location routing protocol is used. Its implementation is more complicated, and there is the problem of frequent switching of routing protocols, which will increase the overhead of the system network and result in poor real-time performance.
5. Routing protocols based on bionic algorithms, such as EGSR (Enhanced Geographical Source Routing) [18], GSO (Glowworm Swarm Optimization) [19], and ASGR (Artificial Spider-Web-Based Geographic Routing) [20]. This type of routing protocol uses a bionic algorithm to select the optimal path to deliver data packets, which can reduce network overhead and end-to-end delay. However, this type of routing protocol is not suitable for high-speed dynamic scenarios.

As can be seen from the above, the latter four routing protocols have the disadvantages of complex algorithm implementation and are not suitable for high-speed mobile Internet of Vehicles. Therefore, this paper studies routing protocols based mainly on the greedy algorithm.

The existing routing protocol based on the greedy algorithm is not perfect, and the following drawbacks exist in its implementation:

- The greedy forwarding strategy has a locally optimal solution when selecting a node. The choice of the next-hop node simply depends on the distance between the judgment node and the target node. There is no global consideration.
- The right-hand rule used when the greedy forwarding strategy fails has drawbacks.
- It does not work well in a sparse network, and can easily fall into a routing hole, resulting in routing death.

In order to solve these shortcomings, a new Weighted-Greedy Perimeter Coordinator Routing (W-GPCR) method is developed in this study to address the following aspects of the GPCR approach:

- The node’s movement direction and density are also taken into consideration, and the optimal next-hop node is selected through weight calculation.
- Through the weight calculation, the direction of data packet delivery will always converge towards the target node, which solves the drawbacks of the right-hand rule.
- Using a restricted forwarding strategy, weight selection can prevent data packets from being delivered again in the direction of routing holes, and find other hidden paths to deliver data packets to target nodes.

## 2. Materials and Methods

The W-GPCR approach is a geographical location routing protocol based on weight selection. It adopts the corresponding adaptive weight parameter ratio for different scenarios to select the optimal next-hop relay node. The application layer of the source node sends data packets to the data link layer, which performs route discovery to obtain sensor data, and sends a RREQ (Route Request) to the next-hop node. The data exchange between the nodes adopts the IEEE802.11p protocol; the GPS module can be used to obtain its position coordinates and the installed IMU (inertial measurement unit) can obtain information such as the node’s movement direction. The next-hop node becomes the current node to execute the same route discovery strategy as the source node, and finally sends the RREQ to the target node. After receiving the RREQ sent by the source node, the target node sends a RREP(Route Reply) according to the optimal path determined by the route discovery process.

When selecting the next-hop node, the traditional greedy forwarding strategy only considers whether the distance between the next-hop node and the target node is smaller than the distance between the current node and the target node. Such a choice can easily cause local optimization problems, but may not be optimal on the global path. Thus, the proposed approach considers the distance between nodes, the driving direction of nodes, and the density of nodes. By calculating the weights, the optimal next-hop node is selected so that the direction of packet delivery will always converge towards the target node, thus avoiding routing loops and other problems. When the next-hop node cannot be found in the signal coverage of the node for packet delivery, the delivery of the data packet falls into the routing hole at this time. In view of such a scenario, a restricted forwarding strategy is proposed to prevent nodes from delivering data packets in the direction of routing holes again and to reduce unnecessary routing overhead.

### 2.1. Greedy Forwarding Strategy Based on Weight Selection

In the existing greedy forwarding strategy, the basis for selecting the next-hop node is the distance between the next-hop node and the target node. This has limitations and can easily cause local optimization problems, so we choose to optimize based on the existing greedy forwarding strategy. Under the premise of judging the distance between the next-hop node and the target node, reference factors are introduced, including the direction of movement and node density of the next-hop node. Instead of simply judging the distance between the next-hop node and the target node, this can reduce the limitations and provide the optimal solution.

#### 2.1.1. Influence of Node Movement Direction on Routing Performance

As shown in Figure 1a, node A sends a data packet to the target node. Node B and node C are closer to the target node than node A. Among these, node C and node A move in opposite directions, while node B and node A move in the same direction. Node C is closer to the target node than node B, so according to the traditional greedy forwarding strategy, node C will be selected as the next-hop node. However, there may be such a situation in which, when the data packet is delivered, the position of the node changes, as shown in Figure 1b. When the data packet is delivered to node C, the next-hop node selected by node C will be node B, which causes extra routing hops. Alternatively, when choosing the next-hop node, we introduce the node movement direction as a reference, instead of relying solely on distance as the basis for selection. When node A selects the next-hop node, it can comprehensively consider the movement direction of node B and node C and their distance from the target node. Selecting node B as the next-hop node will greatly reduce the number of routing hops and shorten the end-to-end delay.

#### 2.1.2. Impact of Node Density on Routing Performance

As shown in Figure 2, node A sends a data packet to target node D. The distances between its neighbors B and C to the target node are the same, but the density of nodes in the signal coverage of node B is greater than that of node C. It can be seen from the figure that if node A forwards the data packet to node B, the subsequent feasibility of establishing a routing path is greater than that of node C. Thus, node density is also one of the important indicators that affect routing performance. The higher the node density, the greater the possibility of routing, and the more likely it is to establish a reliable routing link and improve the delivery rate of data packets.

#### 2.1.3. Weight Calculation of Greedy Forwarding Strategy

Combining the node motion direction and node density, a formula for calculating weights is proposed:

(1) $$G_{n}=g_{1}(1-\frac{D_{nd}}{D_{pd}})+g_{2}\cos(\vec{v_{n}},\vec{l_{nd}})+g_{3}\frac{neig_{n}}{S}$$

where $D_{nd}$ is the Euclidean distance between the next-hop node and the target node in the two-dimensional plane; $D_{pd}$ is the Euclidean distance between the current node and the target node; $\vec{v_{n}}$ is the vector representation of the speed of the next-hop node; $\vec{l_{nd}}$ is the vector representation from the next-hop node to the target node; ${neig}_{n}$ is the number of neighbor nodes in the next-hop node signal coverage; and s is the two-dimensional planar area within the next-hop node signal coverage. The value $1-\frac{D_{nd}}{D_{pd}}$ is used to judge the distance between the next-hop node and the target node. The larger the value $1-\frac{D_{nd}}{D_{pd}}$, the closer the next-hop node is to the target node. The value $\cos(\vec{v_{n}},\vec{l_{nd}})$ is used to judge whether the movement direction of the next-hop node tends to the direction of the target node. The larger the value $\cos(\vec{v_{n}},\vec{l_{nd}})$, the more the movement direction of the next-hop node converges toward the target node. The value $\frac{neig_{n}}{S}$ is used to judge the node density within the signal coverage of the next-hop node. The larger the value $\frac{neig_{n}}{S}$, the greater the possibility of routing. $g_{1},\;g_{2},\;g_{3}$ are the weight ratios of the three reference quantities: $g_{1}$ is the weight ratio of the distance between the nodes, $g_{2}$ is the weight ratio of the node’s movement direction, and $g_{3}$ is the weight ratio of the node density; $g_{1},g_{2},g_{3}\in [0,1]$ and $g_{1}+g_{2}+g_{3}=1$. When the node is far away from the target node, the value $1-\frac{D_{nd}}{D_{pd}}$ will be very small, while the values $\cos(\vec{v_{n}},\vec{l_{nd}})$ and $\frac{neig_{n}}{S}$ will not be greatly affected in this case. In order to weigh the influence of various parameters, we set $g_{1}>g_{2}$ and $g_{1}>g_{3}$ because, under the greedy forwarding strategy, the distance between nodes is used as the main reference quantity, and the movement direction and density of the nodes are used as auxiliary reference quantities.

$G_{n}$ is the weight value of the next-hop node under the greedy forwarding strategy of weight selection. By calculating the weight value of each neighbor node, the neighbor node with the largest weight value will be selected as the next-hop node. The implementation of Algorithm 1 describes the calculation of the weight value and the selection process of the next-hop node.

The notations in Algorithm 1 are shown in Table 1.

When Algorithm 1 is implemented, the neighbor node with the largest weight is selected as the next-hop node.
**Algorithm 1 Pseudo code for W-GPCR**$loc_{p}=getLocation(currentnode)=(x_{p},y_{p})$$\vec{v_{p}}=getSpeed(currentnode)$$neig_{p}=getNeig(currentnode)$$loc_{d}=getLocation(destnode)=(x_{d},y_{d})$$D_{pd}=\sqrt{{\left(x_{p}-x_{d}\right)}^{2}+{\left(y_{p}-y_{d}\right)}^{2}}$$\vec{l_{pd}}=loc_{d}-loc_{p}=(x_{d}-x_{p},y_{d}-y_{p})$$S=\pi r^{2}$$G=g_{2}\cos(\vec{v_{p}},\vec{l_{pd}})+g_{3}\frac{neig_{p}}{S}$nextnode=currentnodefor all neighbors of currentnode do$loc_{i}=getLocation(n_{i})=(x_{i},y_{i})$$\vec{v_{i}}=getSpeed(n_{i})$$D_{i}{}_{d}=\sqrt{{\left(x_{i}-x_{d}\right)}^{2}+{\left(y_{i}-y_{d}\right)}^{2}}$$\vec{l_{i}{}_{d}}=loc_{d}-loc_{i}=(x_{d}-x_{i},y_{d}-y_{i})$$neig_{i}=getNeig(n_{i})$$G_{i}=g_{1}(1-\frac{D_{id}}{D_{pd}})+g_{2}\cos(\vec{v_{i}},\vec{l_{id}})+g_{3}\frac{neig_{i}}{S}$$\mathrm{If}\;G_{i}>G\;\mathrm{then}$$G=G_{i}$$nextnode=n_{i}$end ifend forif. nextnode≠currentnode. thenforward the packet to nextnodeelse carry the packet with currentnodeend if

The system is initialized to obtain the position coordinates, the velocity vector, and the number of neighbor nodes of the current node, and the position coordinates of the target node are also obtained. By calculating the Euclidean distance between the current node from the target node on the two-dimensional plane, and the vector of the current node pointing to the target node the area covered by the signal of the node on the two-dimensional plane can be derived. By calculating the weight of the current node and traversing all of its neighbor nodes, the position coordinates, velocity vector, and number of neighbor nodes of each neighbor node, the Euclidean distance of each neighbor node from the target node and the vector pointing to the target node can be obtained. Based on the obtained data, the weight of each neighbor node is calculated. If the weight of the neighbor node is greater than the weight of the current node, the data packet is sent to the node; otherwise, the current node carries the data packet.

### 2.2. Weight Selection Repair Strategy

When the distance from the current node to the target node is less than the distance from its neighbors to the target node, the greedy forwarding strategy will be invalidated, and the repair strategy will be executed. The traditional repair strategy uses the right-hand rule to deliver data packets, as shown in Figure 3. Node A sends a data packet to node F, traverses its neighbors in a counterclockwise direction according to the right-hand rule, and repeats until the data packet reaches the target node or meets the condition of greedy forwarding to leave the repair strategy. The link path obtained by delivering the data packet according to the right-hand rule in Figure 3 is A-B-C-D-F.

However, in some scenarios, data packets are delivered according to the right-hand rule, and the data packets are delivered far away from the target node. This will result in the unsuccessful delivery of the data packet to the destination, resulting in communication failure. Therefore, the weight calculation formula under the repair strategy is proposed. When the restricted greedy forwarding strategy fails, the data packet is delivered to the intersection node in the street direction. The intersection node will calculate the weights of all neighbor nodes within its signal coverage. By calculating the weights of all neighbor nodes within the signal coverage of intersection nodes, the neighbor node with the highest calculated weight will be selected as the next-hop node, thus solving the problem associated with the right-hand rule.

(2) $$R_{n}=r_{1}(1-\frac{D_{nd}}{D_{pd}})+r_{2}\cos(\vec{l_{pn}},\vec{l_{pd}})+r_{3}\frac{neig_{n}}{S}$$

where $\vec{l_{pn}}$ is the vector representation of the current node pointing to the next-hop node; and $\vec{l_{pd}}$ is the vector representation of the current node pointing to the target node. The value $\cos(\vec{l_{pn}},\vec{l_{pd}})$ is used to judge whether the direction of the selected next-hop node tends to the direction of the target node. A larger value of $\cos(\vec{l_{pn}},\vec{l_{pd}})$ indicates that the delivery direction of the data packet tends to the direction of the target node. $r_{1},r_{2},r_{3}$ is the weight proportion of the three reference quantities: $r_{1}$ is the weight proportion of the distance between the nodes, $r_{2}$ is the weight proportion of the cosine of the packet delivery direction and the target node direction, and $r_{3}$ is the weight proportion of the node density; $r_{1},r_{2},r_{3}\in [0,1]$ and $r_{1}+r_{2}+r_{3}=1$. Under the repair strategy, the distance between the nodes is no longer used as the main reference, but depends on whether the packet delivery direction converges toward the target node. The distance between the nodes and the node density are used as auxiliary references, set as $r_{1}<r_{2}$ and $r_{2}>r_{3}$.

$R_{n}$ is the weight value of the next-hop node under the weight selection repair strategy. By calculating the weight value of each neighbor node, the neighbor node with the largest weight value will be selected as the next-hop node. The calculation of the weight value and the selection of the next-hop node also use Algorithm 1.

As shown in Figure 4, the source node A sends a data packet to the target node H. When the data packet is delivered to the intersection node C, according to the right-hand rule to select the next-hop node, node D will be selected as the next-hop node. The routing path planned by the right-hand rule is A-> B-> C-> D-> E, which will cause the data packet to be delivered away from the target node. According to the weight formula mentioned in this article, $R_{K}<R_{D}$ is obtained through calculation. It can be seen that node K will be selected as the next-hop node, and the repair strategy selected by the weight can plan the routing path of A-> B-> C-> K-> J-> I-> H. The packet is sent to the target node.

### 2.3. Restricted Forwarding Strategy

When a node is forwarding a data packet, it finds that it cannot find the next-hop node for data packet delivery within its signal coverage. This is called the routing hole phenomenon. Routing holes seriously affect normal communication between nodes. In order to avoid communication interruption caused by this phenomenon, a restricted forwarding strategy is proposed. When caught in a routing hole, the node returns the data packet to the intersection node on the street where it reroutes, looking for other paths to deliver the data packet to the target node. In order to avoid rerouting, the data packet is delivered again to the street trapped in the routing hole, and the routing weight calculation formula under the routing hole is proposed:

(3) $$N_{n}=\sin(\vec{l_{in}},\vec{l_{iv}})$$

where $\vec{l_{in}}$ is a vector representation of the intersection node pointing to the next-hop node; and $\vec{l_{iv}}$ is a vector representation of the intersection node pointing to the node trapped in the routing hole. The value $\sin(\vec{l_{in}},\vec{l_{iv}})$ is used to determine whether the direction of packet delivery during rerouting tends to be in the direction of the routing hole. The larger the value of $\sin(\vec{l_{in}},\vec{l_{iv}})$, the less likely the next-hop node selected by the rerouting will fall into the routing hole again.

$N_{n}$ is the weight value of the next-hop node under the restricted forwarding strategy. By calculating the weights of all neighbor nodes within the signal coverage of the intersection node, the neighbor node with the largest weight is selected as the next-hop node for packet delivery.

As shown in Figure 5, the source node O sends a data packet to the target node L. According to the greedy forwarding strategy, when a data packet is delivered to node D, it falls into a routing hole and cannot find the next-hop node to forward the data packet within its signal coverage. At this time, according to the solution proposed in this article, the data packet will fall back to the intersection node C, and node C will reroute to find other paths to deliver the data packet. According to the weight calculation formula in this paper, $N_{E}<N_{F}$ is obtained, so node F will be selected as the next-hop node. Node E will not be selected as the next-hop node, which avoids the dilemma of getting into the empty junction again. After the data packet is delivered to node F, a potential routing path (O-> C-> F-> G-> H-> I-> J-> K-> L) will also be established, which largely guarantees the reliability of normal communication between nodes.

### 2.4. Simulation Model

In this paper, traffic simulation software (SUMO) [21] and discrete network simulation software (NS3) were used to simulate the GPSR, GPCR, and W-GPCR routing protocols in different scenarios. The number of nodes and the source–destination logarithm can evaluate the performance of each routing protocol.

A map of Tianyuan District, Zhuzhou City, Hunan Province was exported from the OpenStreetMap website, as shown in Figure 6a. It was converted into a road file using the netconvert plug-in of SUMO, from which a simulation area of 1000 × 1000 m, and a road traffic model of nine intersections and 12 bidirectional lanes, was selected, as shown in Figure 6b. The initial position of the vehicle was randomly distributed, and the movement of the vehicle on the street was limited by the vehicle following model (i.e., the Krauss model).

Different network conditions were simulated using five different network node numbers: 20, 40, 60, 80, and 100 nodes. Each vehicle was equipped with an omnidirectional antenna and accurate positioning service, which can obtain its position coordinates and driving direction. The communication distance of the vehicle was set to 250 m, and the maximum speed of travel was set to 15 m/s. The MAC(Media Access Control) layer protocol model was set to the IEEE802.11p protocol, the channel transmission rate was set to 3 Mbps, and the transport layer protocol model was set to the UDP(User Datagram Protocol) protocol. The sending interval of the hello packet was set to 1 s, the sending interval of the data packet was set to 0.2 s, and the simulation time was set to 200 s. The data traffic of each node pair (source–destination) was regarded as a constant bit rate (CBR), and a fixed 512-byte data packet was generated by setting a constant bit rate [22,23,24]. The simulation parameters of the model are shown in Table 2.

## 3. Results

In order to evaluate the impact of different amounts of data traffic on the network on routing performance, the number of CBR connections in different node count scenarios was varied between 5, 10, 15, and 20. The weight ratio of the greedy forwarding strategy based on weight selection was set as $g_{1}=0.7$, $g_{2}=0.2$, and $g_{3}=0.1$. The weight ratio of the repair strategy based on weight selection was set as $r_{1}=0.2$, $r_{2}=0.7$, and $r_{3}=0.1$. Through 30 simulation runs, the average values of all simulation data were taken, and a 95% confidence interval was set. Data are finally presented in the form of an error bar graph. The performance indicators used in the simulation are defined as follows:

- Packet delivery rate: the ratio of the total number of packets received by the target node to the total number of packets sent by the source node.
  $$Packet\;deliver\;rate=\frac{N_{receive}}{N_{send}}$$
- Average end-to-end delay: The average delay of all successfully received packets.
  $$Average\;end\text{-}to\text{-}end\;delay=\frac{\sum_{1}^{n}D_{n}}{n}$$
- Average hop: the average number of hops of all nodes in the network.
  $$Average\;hop=\frac{\sum_{1}^{n}H_{n}}{n}$$

### 3.1. Packet Delivery Rate

Figure 7 shows the packet delivery rate of different numbers of nodes and CBR connections. As the number of nodes in the network increases, the connectivity of the network is improved, and the probability of encountering routing holes is reduced. Therefore, with the increase of the number of nodes in the network, the packet delivery rate of these three routing protocols increases. In networks with different numbers of nodes and different CBRs, the packet delivery rate of W-GPCR is higher than that of GPCR and GPSR. In sparse networks with CBR of 10 and 20, and nodes numbering 20, 40, and 60, the packet delivery rate of W-GPCR is much higher than that of GPCR and GPSR. Because the repair strategy of W-GPCR weight selection selects the next-hop node by weight, rather than simply relying on the right-hand rule to traverse the node, routing redundancy is reduced, data packets are prevented from being delivered away from the target node, and the stability of the system is improved.

### 3.2. Average End-To-End Delay

Figure 8 shows the average end-to-end delay for different numbers of nodes and CBR connections. In networks with different numbers of nodes and different CBRs, the average end-to-end delay of W-GPCR is lower than that of GPCR and GPSR. In addition, in the case of the same CBR, the average end-to-end delay of W-GPCR in the network scenario with a differing number of nodes is almost the same. On the contrary, the jitter of GPCR and GPSR is very large. As the number of nodes increases, the average end-to-end delay gradually decreases, and the stability of W-GPCR is stronger than that of GPCR and GPSR. The greedy forwarding strategy selected by the weight of W-GPCR is more global than the greedy forwarding strategy of GPCR and GPSR, which simply considers the distance to the target node. By considering the movement direction and node density of the node, the node with the largest weight among the neighbor nodes is selected as the next-hop node to avoid the packet delivery falling into a local optimum, thus greatly improving the performance of W-GPCR.

### 3.3. Average Hop

Figure 9 shows the average number of hops for different nodes and CBR connections. In networks with a different number of nodes and different CBRs, the average hop count of W-GPCR is less than that of GPCR and GPSR. Because W-GPCR’s restricted forwarding strategy for routing holes in a sparse network provides more routing possibilities, the possibility of successfully delivering data packets to the target node is also greater. W-GPCR can reduce the number of redundant routing hops in the global path of packet delivery, reducing the network overhead of the system.

## 4. Conclusions

The high-speed mobile nodes of the Internet of Vehicles and rapid changes in topology represent significant challenges in designing a routing protocol suitable for VANETs. The W-GPCR routing method proposed in this paper considers the distance from the target node and combines the node’s movement direction and density to design a weight calculation algorithm. In different scenarios of the Internet of Vehicles, the weight parameter ratio is adaptively selected to obtain the optimal next-hop node. The packet delivery rate is used to measure the reliability of routing protocols. The packet delivery rate of the W-GPCR protocol in different networks is higher than that of GPCR and GPSR. By judging whether the delivery direction of the data packet converges toward the target node, the problem caused by the right-hand rule of routing loops traversing the node and being far from the target node is avoided. The end-to-end delay is used to measure the real-time nature of the routing protocol. The end-to-end delay of the W-GPCR routing protocol in different networks is lower than that of GPCR and GPSR. By introducing other reference quantities, such as node movement direction and node density, to select the optimal next-hop node, the delivery of data packets is prevented from falling into a local optimal. The average hop count is used to measure the network bandwidth and time consumed during the packet delivery process. The average hop count of the W-GPCR routing protocol in different networks is less than that of GPCR and GPSR. By judging whether the delivery direction of the rerouted data packet tends to be the direction of the street trapped in the routing hole, the packet delivery is prevented from falling into the routing hole again. In summary, the W-GPCR routing protocol shows better performance than that of GPCR and GPSR in packet delivery rate, average end-to-end delay, and average hops.

## Figures and Tables

**Figure 1:** Schematic diagram of packet delivery: (**a**) before packet delivery; (**b**) after packet delivery.

**Figure 2:** Effect of node density on routing performance.

**Figure 3:** Delivery of data packets according to the right-hand rule.

**Figure 4:** Schematic diagram of the repair strategy for weight selection.

**Figure 5:** Schematic diagram of restricted forwarding strategy.

**Figure 6:** Schematic diagram of the road traffic model: (**a**) map of Tianyuan District, Zhuzhou City, Hunan Province; (**b**) schematic diagram of road files generated by SUMO.

**Figure 7:** Packet delivery rate for varying the number of nodes and constant bit rate (CBR) connections: (**a**) 5 CBR connections; (**b**) 10 CBR connections; (**c**) 15 CBR connections; (**d**) 20 CBR connections.

**Figure 8:** Average end-to-end delay for varying the number of nodes and CBR connections: (**a**) 5 CBR connections; (**b**) 10 CBR connections; (**c**) 15 CBR connections; (**d**) 20 CBR connections.

**Figure 9:** Average hop for varying the number of nodes and CBR connections: (**a**) 5 CBR connections; (**b**) 10 CBR connections; (**c**) 15 CBR connections; (**d**) 20 CBR connections.

**Table 1:** The notations in Algorithm 1.

Notation	Description
currentnode	the current node
nextnode	next-hop node
destnode	target node
$loc_{x}$	the position coordinates of node x
$\vec{v_{x}}$	the velocity vector of node x
$\vec{l_{xd}}$	the vector where node x points to the target node
$neig_{x}$	the number of neighbors of node x
$n_{i}$	the i-th neighbor node
r	the communication radius of the node
getLocation	to get the position coordinates of the node
getSpeed	to get the speed vector of the node
getNeig	to get the number of neighbor nodes

**Table 2:** Simulation parameters.

Parameter	Value
Packet size	512 bytes
Simulation time	200 s
Simulation area	1000 × 1000 m
Bit rate	5, 10, 15, 20
Maximum rate	15 m/s
Number of nodes	20, 40, 60, 80, 100
Hello packet interval	1 s
Transfer Protocol	UDP
Packet interval	0.2 s
MAC layer protocol	802.11p
Channel transmission rate	3 Mbps
Communication distance	250 m
